The article "An Intelligent Supervision for Supply Chain Finance and Logistics Based on Internet of Things" was published in 2022. Journal: Comput Intell Neurosci.

# An Intelligent Supervision for Supply Chain Finance and Logistics Based on Internet of Things

**DOI:** 10.1155/2022/6901601

**Published:** 2022-04-25

**Authors:** Wei Bai, Yongbin Liu, Jingjie Wang

**Affiliations:** Hui Hua College of Hebei Normal University, Shijiazhuang, Hebei 050091, China

## Abstract

Supply chain finance and logistics activities are developing rapidly. In the economic activities of the tripartite cooperation between financial institutions, logistics enterprises, and loan enterprises, the goods will enter the logistics and supervision links of pledged goods immediately after they are postponed. It is proposed to integrate computer network communication technologies such as the Internet of Things with supply chain finance and logistics supervision to strengthen the information interaction between suppliers, which is widely used in supply chain activities to help realize the Internet finance. An intelligent supply chain supervision can implement monitoring and early warning of the time of the pledged goods in the warehouse, in transit, and during processing. Therefore, this paper proposes an intelligent supply chain supervision model by integrating supply chain finance, logistics, and pledge finance models into an operation management platform to better promote the smooth progress of supply chain finance and logistics supervision activities, which can effectively reduce various external risks, improve operational efficiency, and provide reference for supply chain finance and logistics activities.

## 1. Introduction

The concept of supply chain finance originated in the 1980s and developed in the early 21st century, and especially during the financial crisis in 2008, supply chain finance was better developed and applied. From the perspective of the concept of supply chain finance, it emphasizes the integrated services of supply chain management, logistics management, and financial management, involving upstream and downstream suppliers, sellers, logistics suppliers, financial service institutions, etc. of manufacturing and core enterprises [1, 2]. Its basic content is that when the enterprise has insufficient funds, the enterprise will first consider to solve the problem of the funds through the normal credit channel and loan to the financial institution [3]. Under normal situations, financial institutions will ensure the safety of loans by guaranteeing the fixed assets required by the loan unit to avoid risks [4]. However, some small- and medium-sized enterprises cannot obtain financial support from banks because they cannot provide corresponding fixed assets as collateral and thus lose the opportunity to expand reproduction and expansion and even go bankrupt. On the other hand, the competition in the banking industry is becoming more and more fierce, and the traditional loan model can no longer meet the needs of the market, especially some fresh products proposed by new commercial banks, which bring more pressure from market competition. It also needs an innovative business model to design new products to meet the needs of our customers.

Because there are many units involved in supply chain finance, the process is more complicated, and the business models adopted by each unit in the cooperation are different, which leads to different financing requirements and conditions for different enterprises [5]. Rapid development brings some inconvenience and even restricts its development. With the continuous intensification of market competition, behind the rapid development of the financial industry, the supply chain finance business has also shown the drawbacks of product proliferation, high cost, and increased risk due to hasty launch and unfamiliar personnel, which has brought many problems to the majority of banks and employees [6–9]. The three-party logistics enterprises with business supervision have brought unnecessary troubles. Through observation and analysis, it is not difficult to find that, behind the rapid development of supply chain finance, not only the support of core supply chain enterprises and upstream and downstream customers, but also 3PL companies with perfect systems and standardized operations are needed to serve them, so as to jointly meet the health of supply chain finance. In the face of such a huge market gap and virgin land to be developed, as well as the restrictive factors behind the development of supply chain finance in recent years, it is urgent to study the relevant mechanism of supply chain finance business and find out the implementation process of supply chain finance in 3PL enterprises, marketing methods, risk aversion, and other measures to facilitate the healthy, rapid, and lasting development of supply chain finance [10–12].

The concept of the Internet of Things first appeared in the 1990s, and its emergence was produced under the joint action of current Internet technology, network information technology, and logistics monitoring systems [13–15]. In the Internet of Things system, the tracking of related products is realized through the corresponding information transmission and positioning system. Devices and technologies are interconnected through a huge network, so as to realize the information transfer and interaction of data in the network system. In this case, it can ensure the tracking and positioning of information, and at the same time, it can also realize the monitoring and management of information. Therefore, this paper tries to design an intelligent supervision system for supply chain finance and logistics based on Internet of Things. The system improves the authenticity and timeliness of the data in the information system database, reduces manual input errors, and adds a risk rating module to the traditional logistics and warehousing management information system throughout the entire process of activities.

In this paper, the work is organized as follows: In Section 1, the background and motivation are discussed and analyzed. In Section 2, the Internet of Things and supply chain finance techniques are discussed as the basis of this work. In Section 3, an intelligent supervision system for SCM and logistics is designed based on the Internet of Things. In Section 4, some important conclusions and suggestions are performed.

## 2. Internet of Things and Supply Chain Finance

### 2.1. Supply Chain Finance and Logistics

Some scholars have summarized the legal atmosphere, business model, supervision model, and process management of inventory pledge financing [16, 17]. The inventory pledged business model showed new characteristics of reform, and some of its views also had a good enlightenment for the current integration of logistics and finance [18]. Financial resource flows are considered as a financial SCM between logistics and finance, and the management of net current assets is taken as an important research issue under the framework of SCM management [19, 20]. Going beyond the commodity flow optimization scheme based on reducing material inventories, they analyzed the tools of cash management, taking into account the optimal timing of business activities, the control of accounts receivable, liabilities, and prepayments [21]. Pfohl and Gomm [22] used the term SCM finance to refer to the control and optimization of financial flows due to logistics. Hofmann et al. [23] made a theoretical definition of SCM finance: SCM finance is located at the junction of logistics, SCM management, collaboration, and finance and is the a approach in which multiple organizations, including external service providers, jointly create value by planning, directing, and controlling the flow of financial resources between organizations.

Analyzing the operation principles, risk identification, evaluation, and control methods of SCM finance can help 3PL enterprises to discover and apply the blue ocean market of SCM finance, optimize business processes, reduce operating costs, and control risks through a joint marketing mechanism. Using the relevant theories, combined with the application examples of SCM finance in 3PL enterprises, we discuss the relevant laws of 3PL enterprises in developing SCM finance business in the fierce market competition and find out that 3PL enterprises should pay attention to developing SCM finance business vigorously. Combined with the close connection of business flow, logistics, information flow, and capital flow in modern SCM management, it is demonstrated that the application space of SCM finance in 3PL enterprises is very large. It not only brings benefits to financial enterprises' product innovation, but also provides financial enterprises with the logistics enterprises competing in the red ocean bringing a blue ocean market. At the same time, it improves their competitiveness, broadens the product field, and increases the company's income. It is used in the current loan financing of SCM enterprises, pledged storage, transportation and processing of logistics enterprises, and simple financial services. In the supervision of the pledged goods, the warehouse can be divided according to the situation, and the goods can be classified according to the value of the goods, and dynamic supervision and static supervision can also be realized. It is divided into the following two points: (1) The supervision of goods volume is carried out according to the situation of the goods volume. Supervision does a good job in the allocation of warehouses according to the situation. Under normal situations, the independent supervision of a single warehouse means that the collateral is stored in a single warehouse. When the price of the collateral is lower than the warning, the logistics company can notify the company to replenish the goods or add a deposit. Large logistics companies have many warehouses all over the country and even the world. They store their pledges in these warehouses. In this case, they can realize the supervision of the warehouses. However, there are likely to be some other problems in the linkage of multiple warehouses, leading to early warning. There is a problem with the line. The corresponding personnel need to do the corresponding work and at the same time strengthen the supervision of the warehouse to ensure strict supervision. (2) Supervision of goods value: Supervision of goods value refers to tracking the variety, specification, quantity, and quality of the pledged items under the condition that the supervision of the pledged items is not lower than the safety alert and divides them into static pledges and dynamic pledges. Static pledge means that once the materials are handed over to the third-party logistics company during the pledge process, the borrower's materials under pledge before repayment cannot be released from the warehouse, nor can they be replaced at will. Until the borrower repays, the item is always in seizure and cannot be taken out of the warehouse, nor is it allowed to be replaced. The dynamic pledge means that after the pledge is transferred to the warehouse under the supervision of the logistics enterprise, the pledgor can use the replacement pledge that meets the contract requirements according to its own business needs, so as to realize the transaction operation of the goods [24, 25]. The supply chain structure of core business activities is shown in Figure 1. From the supply side to the demand side, it needs to go through three stages: suppliers, enterprises, and users.

The model formula used this time is as follows:

(a) Normalization, i.e., the denominator of Bayesian estimation:
  (1) $$\begin{array}{c} p\left(x|y\right)=\frac{p\left(y|x\right)p\left(x\right)}{\int_{x}p\left(y|x^{\prime }\right)p\left(x^{\prime }\right)dx^{\prime }}. \end{array}$$
(b) Given the joint posterior distribution *f* (*x*, *z*), it is computed:
  (2) $$\begin{array}{c} p\left(x|y\right)=\int_{z}p\left(x,z|y\right)dz\;. \end{array}$$
(c) Expectation
  (3) $$\begin{array}{c} Ep\left(x|y\right)\left(f\left(x\right)\right)=\int_{x}f\left(x\right)p\left(x|y\right)dx. \end{array}$$

Variance is also a type of expectation. There are many aspects of demand forecasting in supply chain uncertainty of Bayesian models.

Based on the given target probability distribution (of high dimensionality), a sample of independent identical distributions is generated, and using the generated samples a discrete approximation of this distribution can be made, where

(4) $$\begin{array}{c} pN\left(x\right)=\frac{1}{N}\sum_{i=1}^{N}\delta_{x^{\left(i\right)}}\left(x\right). \end{array}$$

Among *δ*_(*i*)_(*x*) is Dirac of *x*_*i*_*δ* Function. It is equal to zero at all points except *x*, and its integral over the whole domain is equal to 1. This is an expression for a discrete function. If expressed by a discrete function, it is

(5) $$\begin{array}{c} pN\left(x\right)=\frac{1}{N}\sum_{i=1}^{N}I\left\{x=x_{i}\right\}. \end{array}$$

Then we can use this approximate distribution function to calculate various integrals:

(6) $$\begin{array}{c} I\left(f\left(x\right)\right)=\frac{1}{N}\sum_{i=1}^{N}f\left(x\right). \end{array}$$

However, many distributions are difficult to sample directly, and some methods need to be used, such as rejection sampling, importance sampling, and MCMC. Accept reject sampling is an unknown distribution *p* (*x*), but its upper limit can be known. Then select a well sampled distribution function *q* (*x*) to satisfy

(7) $$\begin{array}{c} p\left(x\right)\leq Mq\left(x\right),\;M<\infty . \end{array}$$

Then the related algorithm calculation is carried out.

Use {*t*_*n*_} to denote the set of times when a sale occurs. Let {*ε*_*t*_^*c*^} be a continuous, piecewise differentiable process suitable for Ft, and let {Δ*t*} be a bounded left continuous process suitable for Ft. *ε*_t_ is decomposed as follows [26]:

(8) $$\begin{array}{c} \varepsilon_{t}=\varepsilon_{t}^{c}+\sum_{t_{n}<t}\Delta t_{n}. \end{array}$$

Constrained constraints on dynamic pricing strategies take the form

(9) $$\begin{array}{c} E\left[{\left(\varepsilon_{t}-\varepsilon_{t\prime }\right)}^{+}g\right]\leq \theta \left(t{}^{\prime }-t\right). \end{array}$$

Discrete approximation:

(10) $$\begin{array}{c} pN\left(x\right)=\sum_{i=1}^{N}\omega \left(x\right)\delta_{x^{\left(i\right)}}\left(x\right). \end{array}$$

Selecting *q* (*x*) to minimize the variance of *f*(*x*)*w*(*x*) can obtain the optimal reference distribution:

(11) $$\begin{array}{c} q\left(x\right)\propto |f\left(x\right)|p\left(x\right). \end{array}$$

The formula for sample standard deviation is

(12) $$\begin{array}{c} s=\sqrt{\frac{\sum_{i=1}^{n}\left(x_{i}-\bar{x}\right)}{n-1}}. \end{array}$$

Among them, *s* is the standard deviation, *x*_*i*_ is the sample data, and *n* is the total number of samples.

### 2.2. The Internet of Things

The Internet of Things is a network application technology that is expanded to the outside world on the basis of the concept and foundation of existing Internet technologies. Its core and foundation are Internet communications, big data, and AI techniques [27–31]. The corresponding users use it to achieve expansion and information exchange. The Internet of Things technology uses radio frequency identification technology to strengthen infrared sensing to achieve global positioning. The application of the system, through the information sensing equipment such as laser scanners, makes the connection between items and the Internet according to the corresponding protocol and realizes the interaction between information, so as to realize intelligent identification and do a good job of positioning, tracking, monitoring, and management. Radio frequency scanning and wireless sensor network are the two core technologies of the Internet of Things. Radio frequency scanning technology can realize comprehensive interactive display, so as to use wireless sensing to obtain the corresponding cargo information collection, integrate the corresponding content into information processing, and automatically identify the goods. The realization of the information exchange of the computer network is embodied in the following aspects: (1) The Internet of Things technology improves the SCM financial logistics activities. The Internet of Things technology mainly includes traditional computer technology and network technology in the SCM financial logistics activities. The communication method realizes interaction, and the analysis is realized through video scanning and wireless sensor technology, so that the corresponding pledged materials can be well prepared, so as to do a good job of scanning the information and ensure the comprehensive analysis of the information. Internet technology and financial logistics information are interconnected, and information network technology is used to associate and match the loan information of customers and bank funds. In the storage and mitigation, loan is mainly based on raw materials, semifinished products, and finished products, so as to achieve financing. (2) The Internet of Things technology reduces the risk of SCM finance and logistics supervision. In SCM finance, loan companies obtain loans from financial institutions and form production and circulation activities, finance procedures in warehouse processing products, and entrust third-party companies to supervise materials that are mortgaged to control the risk of financial logistics activities. Inventory pledge is the main component of material pledge. The pledged goods have strong liquidity, so it is prone to large market changes and fluctuations, which makes it difficult to keep pledges in inventory pledge financing. The first is the production link. The application of Internet of Things technology in the production and manufacturing process can complete the automatic operation of the factory production line and realize the identification and tracking of raw materials and parts on the production line. Infrared sensing technology is to quickly and accurately query the quantity and storage location of raw materials and parts required in the inventory by identifying electronic labels. Secondly, when signing an order, the system generates a unique order number of goods. According to the order, the enterprise's production plan and bill of materials are bound with the order number and associated with the electronic product code, which can monitor the completion of the order in the production process and transportation process in real time. When it comes to the procurement link, the Internet of Things technology is used to number the commodity order and the bill of materials to be purchased, obtain relevant information from the supplier through Internet of Things data exchange, and query or monitor the quantity and production quality of purchased materials at the same time.

SCM finance originates from SCM management and is a branch of SCM management, but it belongs to the category of financial business. It has the following characteristics: It has the characteristics of self-compensation. SCM finance emphasizes that the source of credit repayment is the self-paying trade of the borrowing enterprise; that is, the borrowing enterprise directly uses the loan to repay the loan through the sales revenue. The evaluation conditions of the guaranteed credit are different from the general credit. Banks not only check the customer's credit, but also control the customer's right of goods or related accounts receivable, without paying attention to the customer's fixed assets or the form of guarantee. The SCM finance market belongs to the short-term money market. The account period of SCM finance is generally 3–6 months, which is shorter than the one-year period of ordinary credit loans, and the risk is easier to control. The loan purpose has a more real trade background. SCM finance is a business that borrows the credit of core enterprises to upstream and downstream small- and medium-sized enterprises. As shown in Figure 2, compared with traditional credit business, the guarantee of SCM finance is based on the premise of liquid assets, and financial institutions have to face complex logistics processes. Risks are controlled by controlling the logistics and capital flow of loan companies. Strictly the flow of funds and the whole process of the logistics of loan companies through 3PL are controlled. The characteristics of SCM finance determine the complex relationship of stakeholders in supply chain finance, which also means that the risks of supply chain finance business can be distributed and controlled.

## 3. An Intelligent Supervision System for SCM and Logistics

### 3.1. System Platform Construction

The intelligent supervision system for supply chain finance and logistics operation is built on the basis of Internet of Things to collect, process, and exchange information and support system activities such as the transmission of information on the production and circulation of goods [32–35]. The platform consists of application layer, data integration and interaction layer, and perception operation layer, as shown in the structure diagram of Figure 3.

The subjects involved in supply chain finance include core enterprises, upstream and downstream small- and medium-sized enterprises, financial institutions, and logistics enterprises. Among them, logistics enterprises play an important role in supply chain management and undertake all logistics activities in the supply chain. In supply chain finance, they also act as agents of financial institutions to supervise small- and medium-sized enterprises. This dual identity feature, on the one hand, facilitates financial institutions to conduct credit investigations on loan companies; on the other hand, the overlapping of services and supervision reduces costs and has market pricing advantages for both marketing parties and capital demanders, becoming a favorable condition for market competition. It should be said that supply chain management, to a certain extent, serves as a barrier to pave the way for financial institutions risks and becomes the basic condition for future supply chain finance business. As shown in Figure 4, the relationship between the predicted value and the true value is consistent with the law. With the continuous development of supply chain thinking, the level and ability of supply chain management have also been continuously improved. In this way, the financing credit risk has been reduced, the operational efficiency of supply chain finance has been improved, and the labor cost of operation is reduced.

### 3.2. Supply Chain Finance Logistics Operation with Internet of Things

The most commonly used Internet of Things technology in logistics terminals is QR code and radio frequency scanning. Scanning information is interactively transmitted through wireless sensing technology and Internet technology to ensure real-time monitoring of in-stock materials, accurate quantity and quality of inbound and outbound goods, and quality of goods in transit, to avoid collusion and concealment of information by logistics operators for personal gain; the risk is shown in Figure 5.

Figure 5 shows how changes in various risks are important in the supply system. On the basis of many studies on the Internet of Things to strengthen logistics management by feedback on the status of materials in the warehouse, in transit, and in processing, the Internet of Things, Internet, and computer technology are also used to encrypt the process of supply chain financial logistics information to prevent fake information. Both QR codes and barcodes can realize information duplication and overlay. Compared with barcodes, QR codes can store more information and have a longer storage time. Compared with long-distance scanning labels and scanning equipment, the cost is lower and is being widely used in logistics and other industries. In today's supply chain financial logistics activities, the pledge information transmission is still mainly based on e-mail confirmation. A small number of logistics companies have established their own pledge logistics information platforms, and there are few pledge activities where financial institutions participate in document and process review. Technology Platform: this process requires logistics companies to give financial institutions fully open pledge information, and the platform technology uses electronic label replication technology to help financial institutions such as banks realize electronic document declaration and approval.

Through on-site information acquisition, platform information interaction and integration, and terminal equipment information services such as mobile phones, information systems are designed for the food supply chain in planting and breeding, food processing, distribution, and retail to help supply chain operators control information, identify problems, and provide decision making support. When the price fluctuations caused by the fluctuation of the collateral market, financial institutions, and borrowing companies need to confirm the quantity and quality of the goods, the logistics companies will use the Internet of Things technology to send information on the status of all the collaterals in the warehouse, in transit, and in processing to both the financial institution and the borrowing company. And the three parties will make a shipment or supplement plan according to market changes. Vehicle monitoring mainly relies on positioning system (GPS) and geographic information system (GIS) for handover vehicle positioning and taking pictures, GIS route guidance, refueling positioning, abnormal site positioning monitoring, and information push. In storage, process monitoring mainly depends on RF technology and wireless sensor technology, like Figure 6 changes in the influence of multiple factors. These two Internet of Things technologies simultaneously realize the storage of pledged objects or the transfer of photos in the workshop, monitoring of quantity and status, abnormal alarms, and on-site abnormal processing records. Internet of Things monitoring will automatically generate an alarm when materials in the warehouse, in transit, or in processing are abnormal and notify the three parties; logistics companies should arrive at the site first, confirm site information, make inspection reports, identify problems, and solve them in a timely manner. As shown in Figure 7, credit risk shows a certain pattern. To solve the problem, formulate countermeasures and clarify the responsible person to continue to follow up; after the inspection of the problem, the financial institution and the borrowing company will be notified of the solution; when receiving abnormal information, financial institutions and borrowing company personnel who are qualified to be present should actively participate in the scene. Adjustments and countermeasures are being formulated and implemented.

The supply chain finance business is developing rapidly and vigorously. Because supply chain finance involves a wide range of industries, has huge market potential, and contains huge profits, it not only brings business innovation to the majority of financial institutions, but also solves the problem of small- and medium-sized enterprises by breaking the traditional financing concept of small- and medium-sized enterprises. As Figure 8 shows, changes in various financial risks also have an impact on supply chains. Financing bottlenecks bring huge benefits to supply chain management, as shown in Figure 9, where indicator 4 dominates. Undoubtedly, the birth of supply chain finance business has brought financing convenience to these small- and medium-sized enterprises and promoted the rapid development of the industry. As shown in Figure 10, the overall indicators are stable and there is no huge difference. The huge market demand has also brought a blue ocean market to our country's financial institutions and third-party logistics companies that are in a state of complete market competition.

## 4. Conclusions and Suggestions

Pledge loan information, pledge status supervision information, and pledge status change declaration, approval, and execution information in financial logistics: The three functional modules are integrated into the same information platform, which covers and serves a number of banking and financial institutions, borrowing companies, and logistics supervision companies, optimizes the allocation of resources to a greater extent, and carries out activities such as cofinancing, supervision, and joint storage, transportation, and distribution, to promote the integration of logistics, finance, information, and related services. Supply chain finance and logistics activities use electronic information technology to strengthen their own management operations to ensure supervision, convenience, and safety of entry and exit, so as to grasp market information more comprehensively and accurately. The Internet of Things technology is an effective way to realize operation supervision. It provides a corresponding basis for the current supervision work, so as to realize the transmission and analysis of information content. Supply chain financial logistics activities should be based on third-party honesty, mutual trust and cooperation, and cooperation as the basis. Make corresponding improvements on the basis, solve the current problems through friendly consultation, and ensure that the activities can be carried out smoothly. The Internet of Things technology includes traditional computer technology and Internet technology, as well as two-dimensional code labels, wireless sensing, and radio frequency scanning technology. The corresponding information technology can be combined with hardware and software to realize the application in financial logistics activities, so as to use Internet technology to achieve in the convenient operation of the mobile terminal, the property mortgage can be monitored anytime and anywhere, and the corresponding query work can be done well. Supply chain management technology and on-site management technology are relatively important contents in current logistics management. They can effectively improve the management level and at the same time strengthen the cultivation of personnel quality. Doing a good job in related work can greatly improve the overall strength of the enterprise, thereby promoting the comprehensive development of the enterprise. At present, enterprises should pay attention to the application of informatization and ergonomics, and at the same time, they should strengthen the overall management level, accumulate corresponding experience, and strengthen their own cultural management, through the Internet of Things and Internet electronic information interaction technology to achieve comprehensive improvement, so as to do all the basic work, so as to better improve the storage and transportation of collateral and supervision work, so as to promote the overall development of the enterprise.

## Figures and Tables

**Figure 1:** Supply chain structure diagram.

**Figure 2:** Source of SCM finance risks.

**Figure 3:** Schematic diagram of the structure of the supervision system.

**Figure 4:** True value vs. predicted value by Internet of Things.

**Figure 5:** Value at risk for different strategies.

**Figure 6:** Multifactor influence diagram.

**Figure 7:** Changes in different credit values.

**Figure 8:** Statistical plot of different efficiencies versus certain values.

**Figure 9:** The proportion of indicators.

**Figure 10:** Histogram of changes in risk indicators.

## Data Availability

The data used to support the findings of this study are available from the corresponding author upon request.
